The article "Clinical Pharmacist Intervention on Drug-Related Problems among Elderly Patients Admitted to Medical Wards of Northwest Ethiopia Comprehensive Specialized Hospitals: A Multicenter Prospective, Observational Study" was published in 2022. Journal: Biomed Res Int.

# Clinical Pharmacist Intervention on Drug-Related Problems among Elderly Patients Admitted to Medical Wards of Northwest Ethiopia Comprehensive Specialized Hospitals: A Multicenter Prospective, Observational Study

**DOI:** 10.1155/2022/8742998

**Published:** 2022-07-18

**Authors:** Samuel Berihun Dagnew, Gashaw Binega Mekonnen, Ejigu Gebeye Zeleke, Samuel Agegnew Wondm, Tesfaye Yimer Tadesse

**Affiliations:** ^1^Department of Pharmacy, College of Health Science, Debre Tabor University, Debre Tabor, Ethiopia; ^2^Department of Clinical Pharmacy, School of Pharmacy, College Health Science University of Gondar, Gondar, Ethiopia; ^3^Department of Epidemiology and Biostatistics, Institute of Public Health, College of Medicine and Health Sciences, University of Gondar, Ethiopia; ^4^Department of Pharmacy, College of Health Science Debre Markos University, Debre Markos, Ethiopia

## Abstract

*Background:* Drug therapy in the elderly needs an emphasis on age-related changes in drug pharmacokinetics and pharmacodynamics profile. Hospitalized elderly patients are at risk of more than one disease and polypharmacy associated with these; they are at risk of drug-related problems. This study aimed to assess the role of clinical pharmacy on identifying and resolution of drug-related problems among elderly patients admitted to medical ward of Northwest Ethiopia comprehensive specialized hospitals. *Methods*: A multicenter prospective observational study was conducted. A systematic sampling technique was used. The identified drug-related problem was recorded and classified using Cipolle, and adverse drug reaction was assessed using Naranjo algorithm of adverse drug reaction probability scale, and Medscape was used for drug-drug interaction. Data were analyzed by using STATA software version 14.1. Logistic regression was used, and results were reported as odds ratios (ORs) with 95% Confidence intervals with *P* value < 0.05 statistically significant. *Result*: A total of 389 study participants were included in the study. About 266 (68.4%) of the participants had at least a single drug-related problem. About 503 drug-related problems were identified with a mean of 1.32 (CI: 1.27-1.36) drug-related problem per patient. The three-leading categories of drug-related problems were dose too high 108 (21.5%), nonadherence 105 (20.9%), and adverse drug reaction 96 (19.1%). Alcohol use (AOR = 2.2, 95CI%: 1.23-3.94), source of the drug (AOR = 2.85, 95CI%: 1.63-4.98), length of hospitalization (AOR = 2.32, 95CI%: 1.37-3.95), number of comorbidities (AOR = 1.48, 95CI%: 1.09-1.99), and polypharmacy (AOR = 3.06, 95CI%: 1.72-5.46) were important risk factors for drug-related problems. From the intervention provided, 84.7% were accepted by prescribers. Among the total drug-related problems 67.4% of the problem was totally solved. *Conclusion*: This study revealed that DRPs were high among elderly patients admitted to medical ward of Northwest Ethiopia. Comorbidity, length of hospitalization, ploy-pharmacy, payer, and alcohol drinker were more likely to developed drug-related problems. Treatment optimizations were also done by clinical pharmacists and interventions were well accepted by prescribers.

The article "Clinical Pharmacist Intervention on Drug-Related Problems among Elderly Patients Admitted to Medical Wards of Northwest Ethiopia Comprehensive Specialized Hospitals: A Multicenter Prospective, Observational Study" was published in 2022. Journal: Biomed Res Int.

## 1. Introduction

An absolute increment of the proportion of older populations and getting of illness has become an outstanding demographic trend [1–3]. Older adults are prescribed on average two to five prescription medications with more medications prescribed for those reporting more than one illness [4]. Drug therapy is growing more complex, thus making appropriate patient management increasingly challenging especially for older adults [5]. The number of drug-related problems (DRP) increased with the number of drugs used [6, 7]. A drug-related problem is “an undesirable patient experience that involves drug therapy and that actually or potentially interferes with a desired patient outcome” and that interferes with achieving the expected goals of therapy [8].

Older adults are more than twice as likely to require hospitalization compared with adults in middle age [9]. Comorbidity accompanied by multiple medication use often observed in elderly patients had been associated with several unfavorable outcomes [10]. Those are increase hospitalizations, long-term care admissions, emergency department visits, additional prescriptions, inappropriate medications use, medication non-adherence, drug duplication, drug-drug interactions, higher healthcare costs, and adverse drug reactions [10, 11]. Drugs for older patients have unique challenges since many medications need to be used with special caution because of age-related changes in pharmacokinetics (reduction in renal and hepatic clearance and an increase in the volume of distribution of fat-soluble drugs) and pharmacodynamics [2, 12].

The World Health Organization (WHO) estimates that >50% of all medicines are prescribed, dispensed, or sold inappropriately and more than one half of patients fail to take them properly [13]. In the United States (US), around 200 000 peoples die due to DRPs and cost at least $US 200 billion each year [14]. Thus, drug-related problems lead to substantial morbidity and mortality [15]. The risk of DRPs increases with age and usually increased hospital readmission, morbidity, mortality, and health care costs [6]. A total of 34% to 50% of hospitalized older adults experience poor health outcomes, which can prolong their hospital stay, increase their risk for institutionalization, and increase hospital costs and mortality rates [16]. But pharmaceutical interventions have an average cost savings of $US 1511.0 per case by identified and resolved DRPs [17].

The article "Clinical Pharmacist Intervention on Drug-Related Problems among Elderly Patients Admitted to Medical Wards of Northwest Ethiopia Comprehensive Specialized Hospitals: A Multicenter Prospective, Observational Study" was published in 2022. Journal: Biomed Res Int.

Medication use in elderly accounts for almost one-third of all medication prescribed in the USA. The use of one or more prescription drugs among elder adults had increased from 74% in 1988–1994 to 90% in 2009–2012 [18]. Around two-thirds of Australians over the age of 60 years had use 4 or more drugs [19]. Having more than one disease and polypharmacy are a major problem for elderly patients. It has a major risk factor for prescribing error and adherence problems, ADRs, and other adverse health outcomes [5].

Unresolved DRPs can lead to significant drug-related morbidity or mortality. The impact of clinical pharmacy on clinical and economic outcomes has been addressed in many studies [20]. Appropriate pharmacotherapy can help to minimize the risk of unfavorable outcomes of pharmacotherapy [8]. Treatment optimizations of drug therapy are major strategies to improve good treatment outcomes, reduce expenditure, and potentially save lives. Intervention strategies to improve geriatric pharmacotherapy is targeted at improving the regulatory processes of drug testing, reducing inappropriate prescribing, preventing beneficial drug underuse and use of potentially harmful drugs, and preventing adverse drug interactions [21].

Clinical pharmacy is a health science discipline in which pharmacists provide patient care that optimizes medication therapy and promotes health, wellness, and disease prevention [22]. Pharmacist interventions not only certainly influence patient care but also decrease unnecessary medical outflow [23]. Clinical pharmacists have been shown to improve the usage of high-risk drugs and improve the accuracy of medication regimens in geriatric patients when they do medication reviews [22, 24].

In Ethiopia, there are different studies regarding to DRPs in pediatrics and the adult population. However, those were not interventional, and no studies were conducted among elderly patients particularly in Northwest Ethiopia. Hopefully, this research could be a paramount role in health policymakers, insurers, and other stakeholders in developing policies and guidelines for the prevention and management of DRPs to improve the quality of care.

## 2. Methods

### 2.1. Study Setting, Design, and Period

A multicenter prospective observational study was conducted in Northwest Ethiopia comprehensive specialized hospitals: University of Gondar Comprehensive Specialized Hospital, Debre Tabor Comprehensive Specialized Hospital, Felege Hiwot Comprehensive Specialized Hospital, Tibebe Ghion Comprehensive Specialized Hospital, and Debre Markos Comprehensive Specialized Hospitals from April 30, 2021, to July 30, 2021.

The article "Clinical Pharmacist Intervention on Drug-Related Problems among Elderly Patients Admitted to Medical Wards of Northwest Ethiopia Comprehensive Specialized Hospitals: A Multicenter Prospective, Observational Study" was published in 2022. Journal: Biomed Res Int.

### 2.2. Study Population

Patients aged 60 years and above were admitted to the medical wards of Northwest Ethiopia comprehensive specialized hospital during the data collection period and who fulfill inclusion criteria.

### 2.3. Inclusion Criteria and Exclusion Criteria

Patients of either gender of age 60 years and above who were admitted to the medical ward and took at least one medication and were able to participate in the study were included. Those who have incomplete documented data, patients with hearing, and speaking problems were excluded.

### 2.4. Sample Size and Sampling Technique

The number of patients to be involved in the study is determined by using the single population proportion formula:

(1) $$\begin{array}{c} \text{n}=\frac{\;{\left(Z\alpha /2\right)}^{2}\text{P}\left(1-\text{P}\right)}{d^{2.}}, \end{array}$$

where: *n* = minimal sample size required, *Z* 2 *a*/2 = standard normal deviation at 95% confidence interval corresponding to 1.96, *P* = the probability of DRP on elder event (prevalence), and *d* = the margin of error, a 4% margin of error.

Based on a prospective observational study done at Jimma Hospital, Southwest Ethiopia, the prevalence of DTP was 81.5%, so I take the *P* value from here. Therefore, the *P* value was 0.815%, 𝑍*α*/2 = 1.96, and *d* = 0.04. Therefore, *N* = 362.

After accounting for non-respondents and patients who refused to participate in the study, a final sample size of 398 has been reached.

There are five comprehensive specialized hospitals in Northwest Ethiopia. The sample was allocated based on the patients flow and the bed number of the hospital. Proportional allocation was used to select study subjects based on the number of patients that the respective hospitals contained in their medical wards.

The source population and the sample were *N* = 888 and *n* = 389, respectively.

The interval size *K*:

K = N/n = 888/389 = 2.28 ~ 2.

Sample of each hospital = patient flow each hospital ward∗sample size/source of population

UGCSH = 196∗389/888 = 85.86 ~ 86

DTCSH =167∗389/888 = 73

FHCSH =209∗389/888 = 91.56 ~ 92

TGCSH =145∗389/888 = 63

DMCSH =171∗389/888 = 74.9 ~ 75

The study participants were chosen using systematic random sampling technique. Simple random selection was used to choose the first research participant from one of the two values. Then, every other patient was selected from the patient registration book by selecting elderly patients until the required sample reached from April 30, 2021, to July 30, 2021.

The article "Clinical Pharmacist Intervention on Drug-Related Problems among Elderly Patients Admitted to Medical Wards of Northwest Ethiopia Comprehensive Specialized Hospitals: A Multicenter Prospective, Observational Study" was published in 2022. Journal: Biomed Res Int.

### 2.5. Data Collection Process and Management

The data was collected by using a structured questionnaire adopted from different literature and medical records. The data collection tool was assessed by two senior clinical pharmacists who are academicians and researchers for face validity, completeness, clarity of its contents, and approval obtained. The data collectors were five clinical oriented pharmacists (B.Pharm) who are working at medical ward of Northwest Ethiopia, and the supervisors were four senior pharmacists (2 MSc. in clinical pharmacists and 2 B.Pharm). The collected data were checked out for its completeness during data collection by the principal investigator and supervisors. The principal investigator evaluated the appropriateness of medical therapy using various references such as Beers 2019 Criteria, Dipiro 11 edition, UpToDate 2018, Ethiopian National Guideline on Major NCDs 2016, American diabetic association for diabetes, American college of cardiology (2017 CHF; 2018 blood cholesterol; 2017 HTN), the American Society of Hematology (ASH) (2020 guidelines for the management of venous thromboembolism), and IDSA (2019 pneumonia).

Drug-related problem classification was based on the Cipolle DRP classification. The adverse drug reaction (ADR) probability scale was assessed according to the Naranjo ADR probability scale, Accordingly, ADR probability scale was categorized by taking sum the of 10 questions and grouped as definite, probable, possible, or doubtful if the total score is ≥9, 5–8, 1–4, and 0, respectively, and Medscape was used to check drug-drug interactions. The status of interventions was documented based on Pharmaceutical care network Europe (PCNE) V9.00

A pretest was done on 20 patients before the actual data collection, and some modification (example, income) was considered based on the result of the pretest.

### 2.6. Data Processing and Analysis

Data were cleaned, coded, and entered into Epi data version 4.6.2 software and exported to STATA version 14.1 for further analysis. Categorical variables were described by frequencies and percentages, and continuous variables were described by mean and standard deviation and median and interquartile range after checking the normality of the data. Data were expressed in form of tables, graphs, charts, and texts described based on the characteristics of the data. Binary logistic regression was conducted for each independent variable with the dependent variable to a candidate for multivariable analysis. Variables that pass bivariable logistic regression at the 95% confidence intervals with a *P* value of less than 0.25 were selected to multivariable logistic regression constructed to investigate the associations between these variables and the presence of DRPs. Those variables with a *P* value < 0.05 were considered statistically significant in multivariate analysis. Odds ratio (OR) with 95% confidence interval was also computed for each variable for the corresponding *P* value to show the strength of association; final results were reported as odds ratios (ORs) with 95% CIs.

The article "Clinical Pharmacist Intervention on Drug-Related Problems among Elderly Patients Admitted to Medical Wards of Northwest Ethiopia Comprehensive Specialized Hospitals: A Multicenter Prospective, Observational Study" was published in 2022. Journal: Biomed Res Int.

### 2.7. Operational Definitions

Elders: Even if ages of 65 years are mostly used as the definition of elderly persons in developed countries, the age of 60 is for developing countries [1, 14]

Drug-therapy problem: It is an undesirable event experienced by the patient that involves or is suspected to involve drug therapy and that actually or potentially interferes with desired health outcomes [8]

Adverse drug reaction: Any undesirable event experienced by a patient while taking a medicine, regardless of whether or not the medicine is suspected to be related to the event

Non adherence: When patients do not take their medications as prescribed

Drug interaction: When two or more drugs react with each other may cause to experience an unexpected side effect. Only major drug-drug interaction regimens were reported

Substance use history: It refers to using khat, cigarette, and tobacco within 3 months

Body mass index (in kilograms per square meters): According to WHO, it is interpreted as underweight (BMI < 18.5), normal weight (18.5-24.9), overweight (25.0-29.9), and obese (≥30.0)

Multimorbidity: The presence of two or more diseases

Polypharmacy: According to WHO, ploy-pharmacy is recognized as the use of five or more medications

Interventions: It is the process of a pharmacist identifying and making a recommendation to either to health professionals or patients/caregivers in an attempt to prevent or resolve DRPs [25]

Accepted and fully implemented: When a clinical pharmacist recommendation is accepted by prescribers and therapy modified

Accepted and partially implemented: For example, when the pharmacist recommended starting a drug and this drug was initiated but at a different dose than proposed.

Accepted and not implemented: When the suggestions were recognized and accepted but therapy not changed

Problem partially solved: When the suggested problems were recognized, but the problems not solved during intervention

## 3. Results

About half of the patients (50.9%) out of the 389 study participants were female. The mean (SD) age of the study participants was 69 ± 7.46 years. More than half (57.8%) of the patients were married. Almost two-thirds (67.9%) of the patients were farmers and came from rural areas (71.0%). Over half of the participants (53.2%) received their medication for free (Table 1).

The article "Clinical Pharmacist Intervention on Drug-Related Problems among Elderly Patients Admitted to Medical Wards of Northwest Ethiopia Comprehensive Specialized Hospitals: A Multicenter Prospective, Observational Study" was published in 2022. Journal: Biomed Res Int.

### 3.1. Social Drug and Clinical Characteristics

Regarding to social drug use behavior, 45.2% of patients were taking alcohol. Around three fourths (76.4%) of the patients of body mass index were normal, and the mean (SD) of BMI was 22.5 ± 2.9 kg/m^2^. The median (IQR) GFR were 66.6 (51.6-85.2) ml/min/1.73 m^2^ (Table 2).

### 3.2. Prevalence of Specific DRPs

The three main types of drug-related problems were examined in this study. DRPs were dose too high (21.5%), non-adherence (20.9%), adverse drug reactions (19.1%), need additional drug therapy (14.5%), and dose too low (14.5%) (Table 3).

### 3.3. Adverse Drug Reaction

There were 96 ADRs in all (82 were actual and 14 were potential ADRs). Based on Naranjo probability scale, 41 (50%) patients had probable and 33 (40%), 7 (9%), and 1 (1%) had possible, definite, and doubtful ADR, respectively (Figure 1).

### 3.4. Specific Drugs for ADRs

A total of 82 patients had medication side effects; among the most frequent ADRs were diarrhea/constipation, epigastric pain, skin rash, and bleeding (Table 4).

### 3.5. Drug-Drug Interaction

Only those DDIs that have DRP causes were evaluated in this study. There were discovered 154 DDIs in all. Among these, 93 were dose too high, 47 were dose too low, and 14 potential adverse drug reactions. Omeprazole + clopidogrel, ceftriaxone + heparin, and ceftriaxone + nifedipine were the most common DDIs (Table 5).

### 3.6. Number of DRPs per Patients

A total of 503 DRPs were found in this investigation. Most patients (about 266; 68.38%; CI: 63.74-73.02) experienced at least one drug-related problem. Out of those, 82 (30.843%) patients had two DRPs, 49 (18.42%) patients had three, and 19 (7.14%) patients had four DRPs. The patient's average number of drug-related problems was 1.32 (CI: 1.27 to 1.36) (Figure 2).

### 3.7. Top Eleven Drugs which Were Involved in Specific DRPs

The most frequent drug class involved in DRPs was warfarin, followed by atorvastatin, omeprazole, heparin, ceftriaxone, digoxin, and dexamethasone (Figure 3).

### 3.8. Interventions, Prescriber Acceptance Rate and Outcome of Problem

Pharmacists submitted 493 DRPs for intervention out of a total of 503 that were found, while other healthcare professionals addressed the remaining problems. About a total of 855 interventions were provided at different levels by clinical pharmacists. Nearly half 445(52.0%) of interventions were at the prescriber level, followed by 323 (37.8%) of at drug level and 87 (10.2%) of at patient level. The acceptance rate was calculated based on the interventions proposed and discussed with the prescriber. After discussing with the prescriber of interventions were going to drug level, 39 (12.1%) of the drugs were stopped, 54 (16.7%) of new drugs were started, 79 (24.5%) dosage changed, 25 (7.7) of drugs changed, and 126 (39%) of drugs were monitored. From the proposed, 377 (84.7%) DRPs were accepted. Among total DRPs, about 67.4% of the problems were solved, and 11.5% were partially solved (Table 6).

The article "Clinical Pharmacist Intervention on Drug-Related Problems among Elderly Patients Admitted to Medical Wards of Northwest Ethiopia Comprehensive Specialized Hospitals: A Multicenter Prospective, Observational Study" was published in 2022. Journal: Biomed Res Int.

### 3.9. Factors for the Occurrence of DRPs

Multivariable logistic analysis revealed that patients who paid for their medication had a 2.85 (AOR = 2.85, CI: 1.63-4.98) times higher risk of developing DRPs than those who received it for free. The formation of DRPs in alcohol drinkers by the odds of 2.2 (AOR = 2.2, 95 CI: 1.23 - 3.94) was compared with non-drinkers. Patients who stayed in the hospital for seven days or longer had a 2.32 (AOR = 2.32, CI: 1.37-3.95) times higher chance of developing DRPs than those who stayed for less than seven days. The likelihood that DRPs would develop increases by the odd of 1.48 when there are comorbidities (AOR = 1.48, 95CI percent: 1.09-1.99). Patients who took an average of five or more medicines had a 3.06 (AOR = 3.06; CI: 1.72–5.46) times higher risk of developing DRPs than those who used fewer than five drugs (Table 7).

## 4. Discussion

This study assessed the prevalence and factors contributing to an increased risk of developing one or more DRPs and provided interventions for each DRP among elderly patients admitted to medical wards of Northwest Ethiopia comprehensive specialized hospitals. Drug-related problems are becoming a major public health concern [26]. Due to physiologic changes, several concomitant conditions, an increase in the number of medications, and the complexity of drug regimens, elderly individuals are more at risk of developing DRPs. Therefore, identification and optimization of DRPs in this population is decisive.

In this study, 68.38% of patients had at least one DRP, which is comparable with a study conducted in Northern Sweden 66% [27], but higher than in Canada 41% [28], in Spain 45.1% [26], in Chin 34.5% [29], and in Bangkok 63.3% [30] but lower than the study conducted in India 83.4% [31], Croatia 98.6% [32], the Netherlands 95.9% [6], and Ethiopia 81.5% [33]. The length of the study, the sample size, and the methodology used may all be contributing factors to these variations. Different countries may have very different medical practices and healthcare infrastructure, which can result in a wide range of drug-related problems.

In the current study, dosage too high was the most frequent DRP, followed by non-adherence, adverse medication reactions, and need additional drug therapy, which is comparable with a study conducted in Belgrade [34]. A meta-analysis and systematic study in Ethiopia were shown that need additional drug therapy, low dose, and non-adherence were the most common subtypes of DRPs [35], whereas in a study conducted in the USA, dose too low is the predominated followed by dose too high and needs additional drug therapy and ADR [36]. This is brought on by the changed pharmacokinetics and pharmacodynamics of aged people, in addition to their underlying medical issues. The dose of a drug often impacts the benefits and side effects of the medications.

The article "Clinical Pharmacist Intervention on Drug-Related Problems among Elderly Patients Admitted to Medical Wards of Northwest Ethiopia Comprehensive Specialized Hospitals: A Multicenter Prospective, Observational Study" was published in 2022. Journal: Biomed Res Int.

Finding of contributing factors for DRPs is crucial since it aids in identifying patients who are most vulnerable and need close monitoring of their prescription regimens, and to provide pharmaceutical care interventions. The results of this study revealed that both demographic and clinical characteristics (drug source, alcohol usage, number of diseases, number of drugs, and length of hospitalization) had a statistically significant impact on the development of DRPs.

Accordingly, the source of the drug is one of the risk factors for DRPs, and patients who paid for their medication had a 2.85 times higher likelihood of developing the DRPs, which is in line with a study conducted at Tikur Anbessa specialized hospital [37]. But most studies out of Ethiopia showed that the source of medication is not the risk factor of DRPs. Patients who were taking alcohol about 2.2 times had DRPs. But in a study conducted in Bangkok, there is no statistical difference between a drinker and nondrinker [30]. This could be a result of problems with drug availability, price, and low drug awareness among the general people in Ethiopia.

Patients with one or more medical conditions increased their risk of developing DRPs by 1.48 times when compared to those who did not have any comorbid conditions; this conclusion is consistent with research from the Netherlands [38], India [39], and Norway [40], but differs from a study conducted in Gondar hospital [41] and a multicenter study in southwestern Ethiopian hospitals [42], which is not statistically different. In fact, as comorbidities and the number of medications rise, patients are at a higher risk of getting DRPs.

When compared to patients who did not take polypharmacy, those on polypharmacy experienced DRPs three times more frequently; this result is supported by a study done in the Netherlands [43], in Taiwan [44], Spain [26], and China [29]. Many studies in Ethiopia and outside of Ethiopia have proved that polypharmacy has been highly associated with DRPs. In this fact, polypharmacy is the main risk factor for DRPs because of increased drug-drug interactions, adverse drug reactions, medication errors, non-adherence, and health costs.

The article "Clinical Pharmacist Intervention on Drug-Related Problems among Elderly Patients Admitted to Medical Wards of Northwest Ethiopia Comprehensive Specialized Hospitals: A Multicenter Prospective, Observational Study" was published in 2022. Journal: Biomed Res Int.

Patients who stayed in the hospital for seven or more days were 2.3 times more likely to have DRPs; it is supported by a meta-analysis conducted in Ethiopia [45], a study in China [29], and a multicenter prospective study in southwestern Ethiopia [42]. The reason might be the likelihood of infection in patients who stayed in the hospital for a long time necessitates more management, which raises the expense of patient healthcare.

After identified DRPs, interventions were also made for each DRP. About 855 (98.8%) interventions were provided by clinical pharmacists proposed at three levels: at prescriber, patient level, and drug level. As a result, interventions put forward at the prescriber level were 52.0%, at a patient 10.2%, and drug levels 37.8%, whereas a study in Mangalore showed that interventions at prescriber, at the patient level, and drug level were 77.7%, 26.54%, and 12.32%, respectively [46]; a study in Jimma hospital prescriber level was 40.4% patient/career level 25.7%; and drug level was 33.9% [47]. This difference may be due to the clinical pharmacists who reviewed the DRPs were not integrated into the healthcare team, having no direct involvement with the patient care and did not participate in ward rounds, and the system of the government emphasize towards clinical pharmacy.

Through this investigation, the prescriber's acceptance rate was calculated considering the interventions provided at the prescriber level. Hence, out of 445 interventions provided, 84.7% of them were accepted. This finding was comparable with a study done in Turkey 85.4% [48], and Jimma 81.6% [47], but higher than a study conducted in Spain 74.1% [15] and lower than a study conducted in China 91.9% [28] and in Jimma 91.7% [49]. The variations in acceptance rates could be attributed to the clinical pharmacists' ability to communicate, the mechanism for identifying drug-related problems, and physicians' attitudes about pharmacists.

The outcome of clinical pharmacists' interventions and the status of DRPs were determined. The results of this study show that, of the total number of identified DRPs, 67.4% were fully solved and 11.5% were partially solved, which is in line with research done in Canada [20] and Belgrade [29]. However, this conclusion differs from those in Spain [50] and Mangalore [12]. The difference may be due to the physicians' attitude to pharmacists, and clinical pharmacists strictly follow the status of the problem.

These results cannot be generalized to populations other than those who were admitted to the medical ward because this study solely assesses DRPs among individuals admitted to the medical ward. This circumstance can be considered a limitation of the study

The article "Clinical Pharmacist Intervention on Drug-Related Problems among Elderly Patients Admitted to Medical Wards of Northwest Ethiopia Comprehensive Specialized Hospitals: A Multicenter Prospective, Observational Study" was published in 2022. Journal: Biomed Res Int.

## 5. Conclusion and Recommendation

This study revealed that DRPs were high among elderly patients admitted to the medical ward of northwest Ethiopia. The most prevalent were dose too high, non-adherence, and ADR. Comorbidity, length of hospitalization, ploy-pharmacy, payer, and patients who drink alcohol were more likely to develop DRPs. In addition, treatment optimizations were done by clinical pharmacists, and interventions were well accepted by prescribers. Special preference ought to be given to elder patients who are at a higher risk of developing DRP.

## Figures and Tables

**Figure 1:** ADR status among elderly patients admitted to medical ward of UoGCSH, DTCSH, FHCSH, TGCSH, and DMCSH, Northwest, Ethiopia, 2021.

**Figure 2:** Number of DRP identified from elderly patients admitted to medical wards of UoGCSH, DTCSH, FHCSH, TGCSH, and DMCSH, Northwest, Ethiopia, 2021.

**Figure 3:** Top eleven drugs involved in drug-related problems among elderly patients admitted to medical ward of medical ward of UoGCSH, DTCSH, FHCSH, TGCSH, and DMCSH, Northwest, Ethiopia, 202.

**Table 1:** Socio demographic characteristics of elderly patients admitted to medical ward of UoGCSH, DTCSH, FHCSH, TGCSH, and DMCSH, Northwest, Ethiopia, 2021(*n* = 389).

Variables	Categories	Frequency	Percentage
Sex	Male	191	49.1
	Female	198	50.9
Age	60-74	298	76.6
	≥75	91	23.4
Marital status	Single	31	8.0
	Married	225	57.8
	Divorced	60	15.4
	Windowed	73	18.8
Religion	Orthodox	315	81.0
	Muslim	62	15.9
	Protestant	9	2.3
	Other∗	3	0.8
Educational status	Unable to read and write	280	72.0
	Primary	70	18.0
	Secondary	20	5.1
	College and above	19	4.9
Occupation	Farmer	264	67.9
	Merchant	71	18.2
	Government employee	12	3.1
	Retire	42	10.8
Residence	Urban	113	29.0
	Rural	276	71.0
Source of drug	Payment	182	46.8
	Free	207	53.2

Asterisk (∗) represents Adventists (2) and Atheist (1).

**Table 2:** Social drug and clinical characteristics of elderly patients admitted to medical ward of UoGCSH, DTCSH, FHCSH, TGCSH, and DMCSH, Northwest, Ethiopia, 2021 (*n* = 389).

Variables	Categories	Frequency	Percentage
Social drug use	Alcohol	176	45.2
	Cigarette	19	4.9
	Khat	8	2.1
Renal function, GFR (ml/min/1.73 m^2^)	<30	26	6.7
	30-60	123	31.6
	≥60 Median (IQR) 66.6	240 (51.6-85.2)	61.7
BMI (kg/m^2^)	<18.5	20	5.1
	18.5-24.9	297	76.4
	≥25 Mean (SD) 5.6 ± 2.4	72	18.5
LoH (days)	<7	166	42.7
	≥7	223	57.3
Number comorbidity mean (SD)		2.67 ± 1.09	
Number of drug	<5	139	35.7
	≥5	250	64.3

NB: GFR: glomerular filtration rate; SD: standard deviation filtration rate, BMI: body mass index, LOH: length of hospitalization.

The article "Clinical Pharmacist Intervention on Drug-Related Problems among Elderly Patients Admitted to Medical Wards of Northwest Ethiopia Comprehensive Specialized Hospitals: A Multicenter Prospective, Observational Study" was published in 2022. Journal: Biomed Res Int.

**Table 3:** Type of DRPs identified from elderly patients admitted of UoGCSH, DTCSH, FHCSH, TGCSH, and DMCSH, Northwest, Ethiopia, 2021 (*n* = 503 DRPs).

Types of DRPs	Frequency	Percentage
Dose too high	108	21.5
Non-adherence	105	20.9
ADR	96	19.1
Need additional drug therapy	74	14.7
Dose too low	73	14.5
Unnecessary drug therapy	36	7.1
Infective drug therapy	11	2.2
Total DRPs	503	100

**Table 4:** Drugs which were involved for actual ADR on elderly patients admitted to medical ward of UoGCSH, DTCSH, FHCSH, TGCSH, and DMCSH, Northwest, Ethiopia, 2021.

Drug involved	Types of ADR	Frequency	Percentage
Azithromycin (6¶), morphine (4‡), and ceftriaxone (3¶)	Diarrhea/constipation	13	15.85
Prednisolone (2¶, 2 *ψ*), ferrous sulfate (6‡), hemi-up (1 *ψ*), and warfarin (2 *ψ*)	Epigastric pain	13	15.85
Pyrazinamide (2 *ψ*, 2¶), phenytoin (3†), and propylthiouracil (2¶)	Skin rash	9	13.41
Warfarin (2 *ψ*), heparin (2∗, 3 *ψ*), and aspirin (1 *ψ*)	Bleeding	8	10.98
Captopril (2 *ψ*), furosemide (1¶), vancomycin (1¶), and nifedipine (2∗, 1 *ψ*)	Hypotension	7	4.88
Adrenaline 1 Ω, 2¶,3 *ψ*	Headache	6	7.32
Insulin 3∗, 2 *ψ*	Hypoglycemia	5	6.10
Furosemide 3 *ψ*,2¶	Hypokalemia	5	18.29
Enalapril 4 *ψ*	Acute kidney injury	4	4.8
Hydrochlorothiazide (2¶) and cimetidine (1¶)	Confusion	3	3.66
Dexamethasone 1∗, 2¶	Hyperglycemia	3	
Isoniazid 2¶	Weakness	2	2.44
Diazepam (1¶) and morphine (1 *ψ*)	Depression	2	2.44
Spironolactone 2¶	Hyperkalemia	2	2.44

Note: Ω = doubtful ¶ = possible, *ψ* = probable ∗ = definite.

**Table 5:** Drug-drug interaction among elderly patients admitted to medical ward of UoGCSH, DTCSH, FHCSH, TGCSH, and DMCSH, Northwest, Ethiopia, 2021.

Drugs	Frequency	Severity	Risk of interaction
Atorvastatin + cimetidine	22	Major	Increase the level of anticoagulation
Omeprazole + clopidogrel	18	Major	Decrease effect of clopidogrel
Ceftriaxone + heparin	15	Major	Increase effect of atorvastatin
Warfarin + metronidazole	11	Major	Increase bleeding risk
Cimetidine + clopidogrel	11	Major	Decrease effect of clopidogrel
Warfarin + cimetidine	8	Major	Increase effect of warfarin
Digoxin + nifedipine	7	Significant	Increase the level of digoxin
Azithromycin + heparin	6	Major	Increase effect of heparin
Omeprazole +digoxin	6	Major	Increase risk of digoxin level
Digoxin + azithromycin	6	Major	Increase level of digoxin
Morphine + clopidogrel	6	Major	Decrease effect of clopidogrel
Azithromycin + warfarin	5	Major	Increase effect of warfarin
Warfarin + ciprofloxacin	5	Major	Increase the effect of ciprofloxacin
Aspirin + enalapril	5	Major	Decrease renal function
Enalapril + NPH	5	Significant	Increase effect of insulin
Warfarin + heparin	3	Major	Both increase anticoagulation
Dexamethasone + cimetidine	3	Major	Increase level of dexamethasone
Digoxin + metoprolol	3	Major	Increase risk of braycardia
Cimetidine + hydrocortisone	2	Major	Increase effect of hydrocortisone
Dexamethasone + rifampicin	2	Major	Decrease effect of dexamethasone
Morphine + tramadol	1	Major	Increase dependency
Omeprazole + isoniazid	1	Major	Increase effect of omeprazole
Spironolactone + potassium chloride	1	Major	Risk of hyperkalemia
Omeprazole + rifampicin	1	Major	Decrease effect of omeprazole
Haloperidol + ondansetron	1	Major	Both increase QT interval

The article "Clinical Pharmacist Intervention on Drug-Related Problems among Elderly Patients Admitted to Medical Wards of Northwest Ethiopia Comprehensive Specialized Hospitals: A Multicenter Prospective, Observational Study" was published in 2022. Journal: Biomed Res Int.

**Table 6:** Interventions, prescriber acceptance rate and status of problems on elderly patients admitted to medical ward of UoGCSH, DTCSH, FHCSH, TGCSH, and DMCSH, Northwest, Ethiopia, 2021.

	Interventions	Number	Percentage
Intervention by other		10	1.2
Interventions by pharmacists	Total intervention provided	855	98.8
At prescriber level 445 (52.0%)	Int. proposed and discussed with prescriber	386	86.7
	Prescriber informed only	59	13.3
At patient level 87 (10.2%)	Patient drug counseling	76	87.4
	Spoken to family/care giver	11	12.6
At drug level 323 (37.8%)	Drug stopped	39	12.1
	New drug started	54	16.7
	Dosage changed	79	24.5
	Drug changed	25	7.7
	Monitored	126	39.0
Intervention acceptance rate (at prescriber level) domain *N* = 445			
Int. accepted 377 (84.7%)	Int. accepted and implemented	309	82
	Int. accepted and partially implemented	36	9.5
	Int. accepted but not implemented	32	8.5
Int. not accepted 68(15.3%)	Int. not accepted; no agreement	65	95.6
	Int. not accepted not feasible	3	4.4
Status of the problems (503)			
Problem solved		339	67.4
Prob. partially solved		58	11.5
Problem not solved		106	21.1
	Lack of coordination of prescriber	82	77.4
	No possibility to solve problem	6	5.6
	Lack of coordination of patient	18	17

**Table 7:** Results of a bivariable and multivariable logistic regression analysis of factors associated with DRPs among elderly patients admitted to medical ward of UoGCSH, DTCSH, FHCSH, TGCSH, and DMCSH, Northwest, Ethiopia, 2021.

Variables	Categories	DRPs		COR (95% CI)	∗*P* *value*	AOR (95% CI)	*P* value
		Yes (*n* = 266)	No (*n* = 123)				
Age	60-74	192 (72.2%)	106 (86.2%)	1.00	1	1.00	1
	≥75	74 (27.8%)	17 (13.8%)	2.40 (1.35-4.28)	0.003	1.88 (0.94-3.77)	0.076
Marital status	Single	24 (9.0%)	7 (5.7%)	2.24 (0.93-5.43)	0.073	1.88 (0.65-5.45)	0.244
	Married	136 (51.1%)	89 (72.4%)	1.00	1	1.00	1
	Divorced	50 (18.8%)	10 (8.1%)	3.27 (1.58-6.79)	0.001	1.29 (0.55-3.03)	0.561
	Windowed	56 (21.1%)	17 (13.8%)	2.16 (1.18-3.95)	0.013	1.72 (0.82-3.59)	0.151
Occupational status	Farmer	183 (68.8%)	81 (65.9%)	2.26 (0.71-7.22)	0.169	3.94 (0.90-17.19)	0.068
	Merchant	44 (16.5%)	27 (21.9%)	1.63 (0.48-5.57)	0.436	2.32 (0.50-10.73)	0.283
	Employment	6 (2.3%)	6 (4.9%)	1.00	1	1.00	1
	Retire	33 (12.4%)	9 (7.3%)	3.67 (0. 95-14.15)	0.059	4.23 (0.78-22.87)	0.094
Source of drug	Free	117 (44.0%)	90 (73.2%)	1.00	1	1.00	1
	Payment	149 (56.0%)	33 (26.8%)	3.47 (2.18-5.54)	<0.001	2.85 (1.63-4.98)	<0.001∗
Alcohol	Yes	143 (53.8%)	33 (26.8%)	0.32 (0.20-0.50)	<0.001	2.20 (1.23-3.94)	0.008∗
	No	123 (46.2%)	90 (73.2%)	1.00	1	1.00	1
Cigarette	Yes	18 (6.8%)	1 (0.8%)	8.85 (1.17-67.11)	0.035	4.67 (0.45-48.83)	0.198
	No	248 (93.2%)	122 (99.2%)	1.00	1	1.00	1
Comorbidity mean (SD)		2.67 ± 1.09		1.95 (1.53-2.49)	<0.001	1.48 (1.09-1.99)	0.010∗
Number of drug	<5	62 (23.3%)	77 (26.6%)	1.00	1	1.00	1
	≥5	204 (76.7%)	46 (73.4%)	5.51 (3.47-8.75)	<0.001	3.06 (1.72-5.46)	<0.001∗
LOH (days)	<7	88 (33.1%)	78 (63.4%)	1.00	1	1.00	1
	≥7	178 (66.9%)	45 (36.6%)	3.51 (2.24-5.48)	<0.001	2.32 (1.37-3.95)	0.002∗
GFR (ml/min/1.73 m^2^)	<30	18 (6.8%)	8 (6.5%)	1.29 (0.54-3.08)	0.570	0.86 (0.29-2.51)	0.783
	30-60	96 (36.1%)	28 (22.8%)	1.96 (1.19-3.22)	0.008	1.68 (0.89-3.13)	0.104
	>60	152 (5.1%)	87 (70.7%)	1.00	1		1

NB: GFR: glomerular filtration rate, LOH: length of hospitalization, COR: crude odd ratio; AOR: adjusted odd ratio; CI: confidence interval, *P* value < 0.05, ∗*P* value.

The article "Clinical Pharmacist Intervention on Drug-Related Problems among Elderly Patients Admitted to Medical Wards of Northwest Ethiopia Comprehensive Specialized Hospitals: A Multicenter Prospective, Observational Study" was published in 2022. Journal: Biomed Res Int.

## Data Availability

The data sets used/or analyzed at this study are available from the corresponding author up on reasonable request.

## Abbreviations

ACEI: Angiotensin converting enzyme inhibitors
ADR: Adverse drug reaction
DDI: Drug-drug interaction
DRP: Drug-related problem
DTCSH: Debre Tabor Comprehensive Specialized Hospital
DMCSH: Debre Markos Compressive Specialized Hospital
FHCSH: Felege Hiwot Comprehensive Specialized Hospital
TGCSH: Tibebe Gion Compressive Specialized Hospital
UoGCSH: University of Gondar Comprehensive Specialized Hospital
USA: United States of America
WHO: World Health Organization.
